# Modified Harris Hawks Optimization Algorithm with Exploration Factor and Random Walk Strategy

**DOI:** 10.1155/2022/4673665

**Published:** 2022-04-30

**Authors:** Meijia Song, Heming Jia, Laith Abualigah, Qingxin Liu, Zhixing Lin, Di Wu, Maryam Altalhi

**Affiliations:** ^1^Network Center, Sanming University, Sanming 365004, China; ^2^School of Information and Engineering, Sanming University, Sanming 365004, China; ^3^Faculty of Computer Sciences and Informatics, Amman Arab University, Amman 11953, Jordan; ^4^School of Computer Science, Universiti Sains Malaysia, Penang, Malaysia; ^5^School of Computer Science and Technology, Hainan University, Haikou 570228, China; ^6^School of Education and Music, Sanming University, Sanming 365004, China; ^7^Department of Management Information System, College of Business Administration, Taif University, P.O. Box 11099, Taif 21944, Saudi Arabia

## Abstract

One of the most popular population-based metaheuristic algorithms is Harris hawks optimization (HHO), which imitates the hunting mechanisms of Harris hawks in nature. Although HHO can obtain optimal solutions for specific problems, it stagnates in local optima solutions. In this paper, an improved Harris hawks optimization named ERHHO is proposed for solving global optimization problems. Firstly, we introduce tent chaotic map in the initialization stage to improve the diversity of the initialization population. Secondly, an exploration factor is proposed to optimize parameters for improving the ability of exploration. Finally, a random walk strategy is proposed to enhance the exploitation capability of HHO further and help search agent jump out the local optimal. Results from systematic experiments conducted on 23 benchmark functions and the CEC2017 test functions demonstrated that the proposed method can provide a more reliable solution than other well-known algorithms.

## 1. Introduction

In recent years, because of the low computing cost, simplicity, flexibility, and gradient-free mechanisms [1] and metaheuristic algorithms (MAs) [2–5] have attracted a rising amount of interest. In most cases, MAs are motivated by the ideas of evolution [6–8], human [9–12], animal behavior [13–16], or physics [17–21]. Kennedy et al. [22] inspired by the regularity of flock foraging behavior and proposed particle swarm optimization (PSO) with the characteristics of fast convergence speed and fewer parameters. Mirjalili et al. [23] proposed an algorithm called grey wolf optimization (GWO) based on the grey wolves' hierarchy system and hunting strategies. The whale optimization algorithm (WOA) [24] simulates a whale's random search and predation, bubble attack, and contraction surround behavior. The salp swarm algorithm (SSA) [25] is inspired by the leader guiding followers' behavior of salp swarm chains to food. The sine cosine algorithm (SCA) [26] is proposed to optimize the aircraft wing design problem by searching the image inward or outward with the sine and cosine function, which can deep mine the best position and finally achieves the global optimum. Slime mould algorithm (SMA) [27] is motivated mainly by changes in slime mould morphology during foraging.

In the field of MAs, the no free lunch (NFL) theorem [28] illustrates that there is no one-size-fits-all solution to all optimization challenges. Therefore, many researchers show great interest not only in proposing a new algorithm but also in optimizing classical algorithms.

Zheng et al. [29] propose an algorithm called improved remora optimization algorithm (IROA) that improves the remora optimization algorithm (ROA) by introducing an autonomous foraging mechanism. This mechanism is based on the way the remora finds food on its own. Abualigah et al. [30] combine the arithmetic optimization algorithm (AOA) with SCA's operators for enhancing the local search ability of AOA and verify the effectiveness by some experiments. Jia et al. [31] come up with an algorithm called CMSRSSMA with an improvement of SMA by embedding the composite mutation strategy (CMS) and restart strategy (RS). The CMS aims to enhance the population diversity, and the RS is utilized to avoid the local optima. Liu et al. [32] present a modified remora optimization algorithm (MROA) with Brownian motion and lens opposition-based learning, and it can be suitable for the multilevel thresholding image segmentation application. Meanwhile, the new algorithm introduces the nonlinear escaping energy parameters and random-opposition-based learning strategies to make itself more competitive. Almotairi and Abualigah [33] proposed a method called HRSA, which hybrid the original reptile search algorithm (RSA) and ROA by a novel transition method, and applied it to solving data clustering problems. Zamfirache et al. [34] apply a new algorithm hybrid policy iteration (PI) and GWO algorithm to neural networks and get good results in NN training and solving complex optimization problems. Pozna et al. [35] proposed a new algorithm called PF-PSO that hybrid particle filter (PF) and PSO algorithm and applied the new hybrid method to optimize the position control of the integral-type serve systems.

In 2019, Heidari et al. [36] proposed the HHO algorithm, which is inspired by the Harris hawks' predation behavior in nature, including three stages of exploration, the transformation from exploration to exploitation, and exploitation. HHO has the characteristics of simple principles, fewer parameters, and strong local optimization ability. HHO has been used in the aspect of image segmentation [37], neural network [38], electric machine control [39], and other fields. However, HHO has the weakness of limited optimization accuracy, low convergence speed, and easily jumping into local optimum like other MAs. Therefore, many scholars have improved the HHO algorithm from different perspectives. Ma et al. [40] used the Chan algorithm to calculate the initial solution and replace an individual position to reduce unnecessary exploration and improve the algorithm's convergence speed. Houssein et al. [41] introduced cross and mutation cooperative gene operators and proposed the HHOCM optimization algorithm based on opposition-based learning, which enhanced the ability of exploration and applied it to generate the initial population effectively. Tang et al. [42] introduced the tent chaotic map, an elite hierarchy system, nonlinear escape energy strategy, and Gaussian random walk strategy to improve the convergence speed and accuracy of the algorithm. Jia et al. [43] introduced a mutation strategy and dynamic control parameter for calculating escape energy in the exploration stage and achieved good results by regulating different parameters. The above improvement strategy has improved the performance of the HHO algorithm, but it still has significant room for improvement for the shortcomings of the HHO algorithm.

We proposed the ERHHO algorithm to surmount some weaknesses of the HHO algorithm. Based on different experiments, the proposed algorithm was evaluated with some classic algorithms such as SMA and SSA and some HHO optimizer algorithms such as DHHO and CEHHO. And the results show that the proposed algorithm can perform better than the competitive algorithms and enhance the ability to jump out of the local optimum with minor changes. In particular, this paper made the following main contributions:

- Introduced tent chaotic map to improve the quality of initialized population location
- Proposed the strategy called exploration factor in improving the ability of exploration
- Proposed the random walk strategy to promote the convergence speed and accuracy
- The simulation experiments are tested on 23 standard test functions
- The real-world problems tests are based on CEC2017 test functions and five classical engineering problems

The remainder of this document is structured as follows. A quick summary of HHO is given in Section 2.  Section 3 describes the tent chaotic map, exploration factor, random walk strategy, and ERHHO algorithm. The results and discussion of the proposed algorithm are given in Section 4, which mainly applies to benchmark functions, and real problems include CEC2017 and engineering design problems.  Section 5 contains the conclusions and prospects.

## 2. Harris Hawks Algorithm

The HHO algorithm is motivated by different attack strategies of hawks exploring and attacking their prey. HHO is a population-based optimization technology that consists of three stages: exploration, the transformation of exploration, and exploitation. The different phases of HHO are shown in Figure 1.

### 2.1. Exploration Stage

At this stage, hawks perch in random places based on other members or rabbit locations, which are modeled as follows:

(1) $$\begin{array}{c} X\left(t+1\right)=\left\{\begin{array}{cc} X_{\text{rand}}\left(t\right)-r_{1}\left|X_{\text{rand}}\left(t\right)-2r_{2}X\left(t\right)\right|, & q\geq 0.5,\\ \left(X_{\text{rabbit}}\left(t\right)-X_{m}\left(t\right)\right)-r_{3}\left(LB+r_{4}\left(UB-LB\right)\right), & q<0.5, \end{array}\right. \end{array}$$

(2) $$\begin{array}{c} X_{m}\left(t\right)=\frac{1}{N}\sum_{i=1}^{N}X_{i}\left(t\right), \end{array}$$

where *X*(*t*+1) represents the new position of hawks in the next iteration, *X*_rabbit_(*t*) is the position of prey, and *X*(*t*) is the position of hawks. The modulus means the absolute value of the elements. *r*_1_, *r*_2_, *r*_3_, *r*_4_, and *q* are random numbers in the interval (0, 1). **UB** and **LB** are the upper and lower bounds of variables. *X*_rand_(*t*) is the position of a random hawk population. *X*_*m*_(*t*) is the average location of the current population of hawks.

### 2.2. Transformation of Exploration and Exploitation

The escape energy of the prey is a major factor in the transition stage, which is evaluated with the following equations:

(3) $$\begin{array}{c} E_{1}=2\left(1-\frac{t}{T}\right), \end{array}$$

(4) $$\begin{array}{c} E=E_{0}E_{1}, \end{array}$$

where *t* is the current iteration; *E*_0_ is the initial energy of a prey, varying randomly between −1 and 1; and *T* is the maximum number of iterations.

### 2.3. Exploitation Stage

At this point, the hawks assault the prey using four chasing strategies and the prey's escape behavior. Escaping energy (*E*) and the potential of escape (*r*) are required for a successful capture.

When *r* ≥ 0.5 and |*E*| ≥ 0.5, a soft besiege was conducted by hawks in the following equations, which means the prey has enough energy but gets a failed try for escaping:

(5) $$\begin{array}{c} X\left(t+1\right)=\Delta X\left(t\right)-E\left|JX_{\text{rabbit}}\left(t\right)-X\left(t\right)\right|, \end{array}$$

(6) $$\begin{array}{c} \Delta X\left(t\right)=X_{\text{rabbit}}\left(t\right)-X\left(t\right), \end{array}$$

where Δ*X*(*t*) is the contrast between the position of hawks at iteration *t* and the current position of prey and *X*_rabbit_(*t*) represents the leap strength that changes randomly at each iteration. *r*_5_ is a random number between 0 and 1.

Hawks applies a hard besiege to prey with low escaping energy and fails to escape, which is indicated by *r* ≥ 0.5 and |*E*| < 0.5, modeled as follows:

(7) $$\begin{array}{c} X\left(t+1\right)=X_{\text{rabbit}}\left(t\right)-E\left|\Delta X\left(t\right)\right|. \end{array}$$

When *r* < 0.5 and |*E*| ≥ 0.5, hawks hunt through a smarter soft encirclement called soft besiege with progressive rapid dives, modeled as follows:

(8) $$\begin{array}{c} Y=X_{\text{rabbit}}0v-E\left|JX_{\text{rabbit}}\left(t\right)-X\left(t\right)\right|, \end{array}$$

(9) $$\begin{array}{c} Z=Y+S\times LF\left(D\right), \end{array}$$

where *D* is the problem's dimension, **S** denotes a random vector of size 1 × *D*, and **LF** means the Levy flight function as defined in equations.

(10) $$\begin{array}{c} LF\left(d\right)=0.01\times \frac{u\times \sigma }{{\left|v\right|}^{1/\beta }}, \end{array}$$

(11) $$\begin{array}{c} \sigma ={\left(\frac{\Gamma \left(1+\beta \right)\times \;\sin\pi \beta /2}{\Gamma \left(1+\beta /2\right)\times \beta \times 2^{\beta -1/2}}\right)}^{1/\beta }, \end{array}$$

where **u**, **v** are random normal distribution vector with the size of 1 × *d*, *β* is a constant and bound to a value of 1.5, and Γ is a standard Gamma function. Updating the hawk's positions can be modeled by

(12) $$\begin{array}{c} X\left(t+1\right)=\left\{\begin{array}{c} Y\text{ if }F\left(Z\right)<F\left(X\left(t\right)\right),\\ Z\text{ if }F\left(Z\right)<F\left(X\left(t\right)\right). \end{array}\right. \end{array}$$

When the prey's energy is depleted, a hard besiege is established (*r* < 0.5 and |*E*| < 0.5). The calculation of *Y* and *Z* is modeled as equations (13) and (14). The updating method is as follows:

(13) $$\begin{array}{c} Y=X_{\text{rabbit}}\left(t\right)-E\left|JX_{\text{rabbit}}\left(t\right)-X_{m}\left(t\right)\right|, \end{array}$$

(14) $$\begin{array}{c} Z=Y+S\times LF\left(D\right), \end{array}$$

(15) $$\begin{array}{c} X\left(t+1\right)=\left\{\begin{array}{c} Y\text{ if }F\left(Y\right)<F\left(X\left(t\right)\right),\\ Z\text{ if }F\left(Z\right)<F\left(X\left(t\right)\right). \end{array}\right. \end{array}$$

## 3. Proposed Algorithm

### 3.1. Tent Chaotic Map

For the past few years, many scholars have proved that chaotic maps [44, 45] are capable of improving the search process of a population-based metaheuristic algorithm. In general, chaotic maps are usually introduced into one or several processes such as initial population, exploration, or exploitation stage. The images of the 10 most commonly used chaotic maps are shown in Figure 2.

One of the main purposes of this paper is to enhance the diversity of the initialization population. The initialization of location has a certain influence on the diversity of the population and the stability of the algorithm. HHO algorithm can only guarantee the randomness of the population position at the initialization stage, but randomness does not mean uniformity. The chaotic sequence has certain ergodicity and high randomness. Chaotic mapping can generate random numbers with a uniform distribution between 0 and 1. We tested the listed 10 chaotic maps and verified that tent chaotic map is appropriate to our modified algorithm. The characteristics and randomness of this map can effectively improve the performance by transforming the initial position of hawks. The mathematical description is shown in the following equation:

(16) $$\begin{array}{c} X_{i+1}=\left\{\begin{array}{cc} \frac{X_{i}}{a}, & \text{if }X_{i}<a,\\ \frac{1-X_{i}}{1-a}, & \text{if }X_{i}\geq a. \end{array}\right. \end{array}$$

We enhance the diversity of the initialization population by modifying the initial positions through equation (16), where *X*_*i*+1_ represents the new position of hawks after chaotic mapping, *X*_*i*_ is the current position of hawks, and *a* is set to 0.7.

### 3.2. Exploration Factor

In the exploration stage, the HHO algorithm updating positions is mainly calculated by equations (1) and (2), where *r*_1_ and *r*_3_ are random values in the range of (0, 1). Although the settings could lead to the randomness of each step in the global search, the variability is lacking.

In this phase, the original HHO algorithm simulates the situation that the hawks can track and detect the prey with their powerful eyes, but occasionally, the prey cannot be seen easily, and the hawks detect a prey maybe after several hours. According to these, we think we should adjust the parameters to be more flexible.

We can consider the parameters of *r*_1_ and *r*_3_ as the step length; when the values are bigger, the hawks move faster and vice versa. There are two possibilities for a hawk finding a prey, one is an immediate detection, and another is a long-time search. For the first situation, we should consider the randomness of the step length. And, for the second situation, the whole variant trend of the step length should decrease. Because the possibility for a hawk finding a prey increases as time goes by, the hawks should explore a wider range with a bigger step at first, and a meticulous search should be applied in the late iterations. Thus, we update *r*_1_ and *r*_3_ by exploration factor modeled as follows:

(17) $$\begin{array}{c} ef=\left(b\times \text{rand}\left(\right)-\frac{b}{2}\right)\times \;\cos\left(\frac{\pi }{2}\times {\left(\frac{t}{T}\right)}^{2}\right). \end{array}$$

Then equation (1) is updated as follows:

(18) $$\begin{array}{c} X\left(t+1\right)=\left\{\begin{array}{cc} X_{\text{rand}}\left(t\right)-ef\left|X_{\text{rand}}\left(t\right)-2r_{2}X\left(t\right)\right|, & q\geq 0.5,\\ \left(X_{\text{rabbit}}\left(t\right)-X_{m}\left(t\right)\right)-ef\left(LB+r_{4}\left(UB-LB\right)\right), & q<0.5, \end{array}\right. \end{array}$$

where *b* is set to 2 that can achieve a pleasing effect through experimental tests. (*b∗*rand() − *b*/2) is introduced to gain the randomness of step length by generating random numbers in the interval of (−*b*/2, *b*/2). The cos function is introduced to form a nonlinear convergence from 1 to 0 with iterations (see Figure 3).

In a word, the exploration factor expands the range of step length from (0, 1) to (−*b*/2, *b*/2) at first and helps the exploration process gradually change from an extensive range to a small range as the number of iterations increases (see Figure 4). Finally, the exploration factor preserved the randomness of step length.

### 3.3. Random Walk Strategy

In the exploitation stage of the HHO algorithm, Harris hawks update its position through four pursuit strategies. Although it increases the possibility of exploration, entering the next iteration without interference can easily lead to the algorithm falling into the local optimum. To ameliorate this problem, some common strategies are applied to the methods, such as the Gaussian random walk strategy [42], Levy flight function, and Brownian motion [16, 46]. These strategies possess the traits of stabilizing in a range of values with high probability and drastic changing values with low probability. And all these strategies improve the methods by generating a deviation.

In this paper, we think that in the early iterations, the deviation should be bigger so that we can get more chances to jump out of local optima. In the late iterations, a smaller deviation can help find the optimal result better. So we designed the step of random walk gradually taper with iterations. According to these, the random walk strategy was proposed, which is activated by identical fitness values in iterations. In other words, when the value of fitness is equal to its last iteration, we activate the random walk strategy. This strategy can deviate the position of a hawk according to a varying parameter. The value of the parameter depends on (*c* × rand() − *c*/2) × cos(*π*/2 × (*t*/*T*) and decreases with iterations. The strategy is modeled as follows:

(19) $$\begin{array}{c} X_{m}\left(i\right)=X\left(i\right)+\;\left(c\times \text{rand}\left(\right)-\frac{c}{2}\right)\times \;\cos\left(\frac{\pi }{2}\times {\left(\frac{t}{T}\right)}^{2}\right)\times \left(X\left(i\right)-X_{\text{rabbit}}\right). \end{array}$$

When *c* = 6, we can obtain a better performance through the experimental test. *X*_*m*_(*i*) is the new position after applying the random walk strategy. We retain the better result to enter the next iteration by greedy strategy modeled as follows:

(20) $$\begin{array}{c} X\left(t+1\right)=\left\{\begin{array}{cc} X_{m}\left(t+1\right), & f\left(X_{m}\left(t+1\right)\right)<f\left(X\left(\right)\left(t+1\right)\right),\\ X\left(t+1\right), & f\left(X_{m}\left(t+1\right)\right)\geq f\left(\left.X\right)\left(\left(t+1\right.\right)\right). \end{array}\right. \end{array}$$

### 3.4. The Details of ERHHO

HHO possesses strong local exploitation ability but insufficient global exploration. The switch from exploration to exploitation is based on the prey's escaping energy. The population diversity is insufficient in the early iterations, reflecting the exploration period and the slow convergence speed. The energy of prey drops as the number of iterations grows, and the algorithm enters the period of local exploitation. Four different hunting techniques are applied based on the prey's energy and the likelihood of escaping.

Therefore, the tent chaotic map was introduced to enhance the population diversity; then, we optimized critical parameters in the exploration phase with the exploration factor. As a component of the exploitation phase, a random walk strategy was introduced to enhance the ability to jump out of local optima. The convergence speed and accuracy are improved through all of these approaches, and the program's overall optimization performance is effectively enhanced. This new Harris hawks optimization algorithm is called ERHHO.  Figure 5 depicts the summary flowchart, and Algorithm 1 represents the pseudocode for ERHHO.

### 3.5. Computational Complexity Analysis

Initialization, position updating, and fitness evaluation are the three essential components of ERHHO. Positions are generated with a computational complexity of *O*(*N* ∗ *D*), where *N* denotes the number of populations and *D* represents the dimensions of the problem. It takes *O*(*N*) to evaluate the fitness solution. We employ a random walk strategy to prevent the algorithm from entering local optima, and the computational complexity is *O(*2 × *N* × *D* × *T*). Hence, the proposed ERHHO algorithm has a total computational complexity of *O*(2 × *N* × *D* × *T*).

## 4. Experimental Results and Discussion

In this part, we validate the performance of ERHHO on 23 benchmark functions [47] by comparing it with some state-of-art metaheuristics algorithms: SMA, WOA, SSA, SCA, and HHO, and HHO-based optimization algorithm: DHHO/M and HHOCM. Meanwhile, we use the Wilcoxon signed-rank test to acknowledge the differences between ERHHO and the comparative algorithms. Furthermore, we test ERHHO with HHO-related algorithms: HHO, DHHO/M, HHOCM, and CEHHO on CEC2017 test functions to testify the real-world applications. And also the five engineering design issues are applied with the same algorithms as in benchmark functions' tests.

### 4.1. Benchmark Functions and Parameter Settings

Many scholars employ benchmark functions. Details of the unimodal, multimodal, and fixed-dimension multimodal benchmark functions are shown in Table 1. The unimodal benchmark functions (F1–F7) have only one extreme point; it can be effectively testified to the exploitation ability of ERHHO. And the global search capacity of ERHHO can be tested by the multimodal benchmark functions (F8–F23) with many local optima.

To make the experimental findings more representative, the ERHHO is compared with algorithms of SMA [27], WOA [24], SSA [25], SCA [26], and HHO [36], DHHO/M [43], and HHOCM [41].  Table 2 shows the parameter settings for each algorithm. All the parameters are set according to the original articles except *b* and *c* (the analysis of *b* and *c* are listed in Section 4.2). The maximum iteration (*T*) was set to 500; the population size (*N*) was set to 30; and the dimension size (*D*) was set to 30 in all tests. We calculate average results and standard deviations with 30 independent runs and bold the best values.

### 4.2. Sensitivity Analysis of *b* and *c* on ERHHO

The parameter settings of comparative algorithms are in accordance with the original articles, as well as the values of *β* and *a* of ERHHO are according to the original HHO algorithm. The new parameters are *b* and *c*, which can significantly impact the performance of ERHHO. Thus, setting the appropriate parameters for better results is necessary. The aims of *b* and *c* are to find a suitable search range. According to equation (17), the original range is between 0 and 1; for expanding the scope, *b* is considered as 2, 4, and 6; and *c* is considered as 2, 4, and 6. To find the fit *b-c* value pair, we tested 9 situations by using 23 benchmark functions. We calculate the mean results of each function with 30 independent runs, and the results are listed in Table 3. The lowest values are highlighted in bold. We count the number of bold fonts in each function, and the ERHHO algorithm can get the best performance with *b* = 2 and *c* = 6. The parameter values will be used for further experimental tests.

### 4.3. Analysis of Benchmark Functions

#### 4.3.1. Numerical Analysis

For the unimodal benchmark functions (F1–F7), ERHHO can obtain the best result except for F6 as shown in Table 4. Especially, for F1–F4, ERHHO can obtain the theoretical optimum. And the result of ERHHO ranks only second to SSA for F6. The aim of unimodal benchmark functions is to measure the exploitation ability. From the experimental tests of F1–F7, we can prove that the proposed algorithm possesses a strong local search ability.

For the multimodal functions (F8–F23), ERHHO gets the best mean values except for F9 and the best stand deviations except for F14 and F20. The goal of multimodal functions is to evaluate the exploration capability. From the test of F8–F23, we can verify that the global ability of ERHHO is excellent.

In conclusion, the ERHHO algorithm outperforms the other compared algorithms in unimodal functions, which due to the random walk strategy, the algorithm's capacity to jump out of the local optimum can be effectively boosted. For the multimodal benchmark functions, the performance of proposed ERHHO is competitive as well. The reason for the excellent performance of ERHHO in the exploration phase is mainly due to the exploration factor. The exploration factor can expand the scope of exploration that is why ERHHO can find the result faster and more accurately. We tried the experiment of adding the exploration factor only to the original HHO, and the results of some multimodel test functions were better than before. Especially, for F21–F23, the result was improved remarkably and close to the theoretical values (see Table 5).

#### 4.3.2. Convergence Analysis

Figure 6 depicts the results of analyzing the proposed algorithm's convergence in various functions (F3, F5, F7–F10, F12–F15, and F19–F23). For unimodal functions (F3, F5, and F7), the differences in convergence curves between ERHHO and HHO can be observed visually from F5, which represents higher accuracy values after several step-like descents. That is, because when the hawks get trapped, ERHHO activates the random walk strategy, which can help the hawks fly deviate from the trap and lead to a new position with more possibilities. These three functions can reflect that ERHHO possesses a faster convergence speed and a higher accuracy than HHO and the other competitive algorithms in unimodal functions.

The conclusion also holds in multimodal functions. Many of the figures show the ERRHO can get the optimal values directly after several iterations such as F8–F10, F14–F15, and F19–F23 that is because of the strong exploration ability of ERHHO whose global search scope is twice as wide as before in the early period, so the ERHHO algorithm can converge very fast. For F12, the ERHHO and HHO get a similar trend before iteration 100, but after that, ERHHO dive suddenly and get the best accuracy from all competitors. The reason is the coordination of local strategy and global search ability. The local strategy has the characteristic of a large deviation in the early stage and a small deviation in the later period. The cooperation helps the ERHHO jump out of the local optima and find better fitness values by a wide search scope. The situation is reflected in F13 as well because the functions of F12 and F13 have similar graphical features (many close local optimal points).

It can be seen that no matter for unimodal functions or multimodal functions, the proposed algorithm provides a better convergence pattern in almost all functions.

### 4.4. Wilcoxon Signed-Rank Test

The Wilcoxon signed-rank (WSR) test is used to show that the results are statistically significant. By WSR, we can determine whether two sets of values are significantly different. A *p* value is lower than 0.05 suggests that the method is considerably better than the compared algorithms. The Wilcoxon signed-rank test results for each benchmark function are shown in Table 6. As can be observed, ERHHO outperforms almost all of the other algorithms to varying degrees.

### 4.5. The Performance of ERHHO on the CEC2017

To further evaluate, one of the most challenging test functions is called CEC2017 [48], which includes 30 test functions with unimodal, multimodal, hybrid, and composition types (see Table 7). In this experiment, we set dim = 10 for all functions.

HHO algorithm performs poorly on complicated problems such as CEC2017 but focuses on tackling simple, traditional, high-dimensional issues. We compared the proposed algorithm with HHO or optimizer based on HHO is more rational. We tested ERHHO on CEC2017 test functions (excluding F2, which is unstable) and compared it with HHO, DHHO/M, HHOCM, and CEHHO [42]. Each function was put to the test 30 times with 1,000 iterations, and the dimensions of all functions were set to 10.

The results of CEC2017 test functions are listed in Table 8, which utilize Friedman's mean rank, and the best values are provided in bold. According to Table 8, the proposed algorithm performed well in F1 and got the second rank in F3. We can say, the performance of ERHHO is similar to HHOCM and better than other algorithms for unimodal functions. For multimodal functions, ERHHO has a slight advantage over HHOCM and CEHHO but outperforms others. But, for hybrid and composition functions, ERHHO shows a huge lead over the other algorithms. We evaluate the algorithms group by different types of unimodal, multimodal, hybrid, and composition (see Figure 7). From Figure 7, ERHHO got the same Friedman rank value as HHOCM on the type of unimodal and multimodal but obviously outperformed other algorithms. For the type of hybrid and composition, ERHHO got the optimal ranking in all competitive algorithms.

### 4.6. Experiments on Engineering Design Problems

We analyze the performance of ERHHO on five classic engineering design issues in this section. We perform all the experiments by setting the population (*N*) to 30 and the maximum iteration (*T*) to 500. The proposed algorithms are compared to algorithms: SMA, WOA, SSA, SCA, HHO, DHHO/M, and HHOCM. The parameter settings are identical to those listed in Table 2.

#### 4.6.1. Tension/Compression Spring Design Problem

This challenge [49] aims to find the optimum variables of wire diameter (*d*), average coil diameter (*D*), and the number of active coils (*N*) by the optimization algorithms for obtaining the minimum weight of the tension or compress spring under four constraints. The tension/compression spring structure is shown in Figure 8. The conditions and formulations are as follows:

Consider

(21) $$\begin{array}{c} \overset{⟶}{x}=\left[x_{1}\;x_{2}\;x_{3}\;x_{4}\right]=\left[dDN\right]. \end{array}$$

Minimize

(22) $$\begin{array}{c} f\left(\overset{⟶}{x}\right)=\left(x_{3}+2\right)x_{2}x_{1}^{2}. \end{array}$$

Subject to

(23) $$\begin{array}{c} g_{1}\left(\overset{⟶}{x}\right)=1-\frac{x_{2}^{3}x_{3}}{71785x_{1}^{4}}\leq 0,\\ g_{2}\left(\overset{⟶}{x}\right)=\frac{4x_{2}^{2}-x_{1}x_{2}}{12566\left(x_{2}x_{1}^{3}-x_{1}^{4}\right)}+\frac{1}{5108x_{1}^{2}}\leq 0,\\ g_{3}\left(\overset{⟶}{x}\right)=1-\frac{140.45x_{1}}{x_{2}^{2}x_{3}}\leq 0,\\ g_{4}\left(\overset{⟶}{x}\right)=\frac{x_{1}+x_{2}}{1.5}-1\leq 0. \end{array}$$

Variable range

(24) $$\begin{array}{c} 0.05\leq x_{1}\leq 2.00,\\ 0.25\leq x_{2}\leq 1.30,\\ 2.00\leq x_{3}\leq 15.00. \end{array}$$

Table 9 shows the results of ERHHO and compared algorithms for solving this problem, and we can see that the ERHHO algorithm obtained the best performance among all competitors.

#### 4.6.2. Pressure Vessel Design Problem

The problem's primary goal is to obtain set values of the shell (*T*_*s*_), the thickness of the head (*T*_*h*_), the inner radius (*R*), and the length of the cylindrical section (*L*) by the optimization algorithms for reducing the cost of cylindrical pressure vessels [51] while meeting the pressure requirements. The structure of the pressure vessel is shown in Figure 9. The mathematical formula is represented as follows:

Consider

(25) $$\begin{array}{c} \overset{⟶}{x}=\left[x_{1}x_{2}x_{3}x_{4}\right]=\left[T_{s}T_{h}RL\right]. \end{array}$$

Minimize

(26) $$\begin{array}{c} f\left(\overset{⟶}{x}\right)=0.6224x_{1}x_{3}x_{4}+1.7781x_{2}x_{3}^{2}+3.1661x_{1}^{2}x_{4}+19.84x_{1}^{2}x_{3}. \end{array}$$

Subject to

(27) $$\begin{array}{c} g_{1}\left(\overset{⟶}{x}\right)=-x_{1}+0.0193x_{3}\leq 0,\\ g_{2}\left(\overset{⟶}{x}\right)=-x_{3}+0.00954x_{3}\leq 0,\\ g_{3}\left(\overset{⟶}{x}\right)=-\pi x_{3}^{2}x_{4}-\frac{4}{3}\pi x_{3}^{3}+1296000\leq 0,\\ g_{4}\left(\overset{⟶}{x}\right)=x_{4}-240\leq 0. \end{array}$$

Variable range

(28) $$\begin{array}{c} 0\leq x_{1}\leq 99,\\ 0\leq x_{2}\leq 99,\\ 10\leq x_{3}\leq 200,\\ 10\leq x_{4}\leq 200. \end{array}$$

We can see from Table 10 that ERHHO was able to find the optimal solution at the lowest cost compared to other competitor algorithms.

#### 4.6.3. The Three-Bar Truss Design Problem

The three-bar truss design problem arises from civil engineering [52, 53]. This problem aims to minimize the weight in truss design with stress, deflection, and buckling constraints. There are two parameters, *A*1 and *A*2, involved in this design problem, and we should find the best value of *A*1 and *A*2 by the optimization algorithm for achieving the goal above. The design is shown in Figure 10. The model of the problem is depicted as follows:

Consider

(29) $$\begin{array}{c} \overset{⟶}{x}=\left[x_{1}\;x_{2}\right]=\left[A_{1}\;A_{2}\right]. \end{array}$$

Minimize

(30) $$\begin{array}{c} f\left(\overset{⟶}{x}\right)=\left(2\sqrt{2}x_{1}+x_{2}\right)\times l. \end{array}$$

Subject to

(31) $$\begin{array}{c} g_{1}\left(\overset{⟶}{x}\right)=\frac{\sqrt{2}x_{1}+x_{2}}{\sqrt{2}x_{1}^{2}+2x_{1}x_{2}}P-\sigma \leq 0,\\ g_{2}\left(\overset{⟶}{x}\right)=\frac{x_{2}}{\sqrt{2}x_{1}^{2}+2x_{1}x_{2}}P-\sigma \leq 0,\\ g_{3}\left(\overset{⟶}{x}\right)=\frac{1}{\sqrt{2}x_{2}+x_{1}}P-\sigma \leq 0. \end{array}$$

Variable range

(32) $$\begin{array}{c} 0\leq x_{1},x_{2}\leq 1. \end{array}$$

The results for the three-bar truss design problem are listed in Table 11. As we can see, the ERHHO algorithm can achieve the best performance as well as the SSA algorithm in solving this problem.

#### 4.6.4. Cantilever Beam Design

Cantilever beam design is one problem in which hollow square cross-section parameters (*x*_1_–*x*_5_) are optimized [54] by optimization algorithms to obtain the cantilever beam's minimum weight. This problems' architecture is depicted in Figure 11. The mathematical equations are described as follows:

Consider

(33) $$\begin{array}{c} \overset{⟶}{x}=\left[x_{1}x_{2}x_{3}x_{4}x_{5}\right]. \end{array}$$

Minimize

(34) $$\begin{array}{c} f\left(\overset{⟶}{x}\right)=0.6224\left(x_{1}+x_{2}+x_{3}+x_{4}+x_{5}\right). \end{array}$$

Subject to

(35) $$\begin{array}{c} g\left(\overset{⟶}{x}\right)=\frac{60}{x_{1}^{3}}+\frac{27}{x_{2}^{3}}+\frac{19}{x_{3}^{3}}+\frac{7}{x_{4}^{3}}+\frac{1}{x_{5}^{3}}-1\leq 0. \end{array}$$

Variable range

(36) $$\begin{array}{c} 0.01\leq x_{1},x_{2},x_{3},x_{4},x_{5}\leq 100. \end{array}$$

Table 12 summarized the findings, from which we can see that ERHHO was capable of finding the optimal solution and obtained total weight is minimized.

#### 4.6.5. Speed Reducer Problem

The speed reducer problem [55] aims to minimize the reducer's weight by optimizing seven variables *x*_1_–*x*_7_ through the optimization algorithms. The structure of this problem is depicted in Figure 12. The formulas and constraints are written as follows:

Minimize

(37) $$\begin{array}{c} f\left(\overset{⟶}{x}\right)=0.7854x_{1}x_{2}^{2}\left(3.3333x_{3}^{2}+14.9334x_{3}-43.0934\right),\\ -1.508x_{1}\left(x_{6}^{2}+x_{7}^{2}\right)+7.4777\left(x_{6}^{3}+x_{7}^{3}\right). \end{array}$$

Subject to

(38) $$\begin{array}{c} g_{1}\left(\overset{⟶}{x}\right)=\frac{27}{x_{1}x_{2}^{2}x_{3}}-1\leq 0,\\ g_{2}\left(\overset{⟶}{x}\right)=\frac{397.5}{x_{1}x_{2}^{2}x_{3}^{2}}-1\leq 0,\\ g_{3}\left(\overset{⟶}{x}\right)=\frac{1.93x_{4}^{3}}{x_{2}x_{3}x_{6}^{4}}-1\leq 0,\\ g_{4}\left(\overset{⟶}{x}\right)=\frac{1.93x_{5}^{3}}{x_{2}x_{3}x_{7}^{4}}-1\leq 0,\\ g_{5}\left(\overset{⟶}{x}\right)=\frac{\sqrt{{\left(745x_{4}/x_{2}x_{3}\right)}^{2}+16.9\times 10^{6}}}{110.0x_{6}^{3}}-1\leq 0,\\ g_{6}\left(\overset{⟶}{x}\right)=\frac{\sqrt{{\left(745x_{4}/x_{2}x_{3}\right)}^{2}+157.5\times 10^{6}}}{85.0x_{6}^{3}}-1\leq 0,\\ g_{7}\left(\overset{⟶}{x}\right)=\frac{x_{2}x_{3}}{40}-1\leq 0,\\ g_{8}\left(\overset{⟶}{x}\right)=\frac{5x_{2}}{x_{1}}-1\leq 0,\\ g_{9}\left(\overset{⟶}{x}\right)=\frac{x_{1}}{12x_{2}}-1\leq 0,\\ g_{10}\left(\overset{⟶}{x}\right)=\frac{1.5x_{6}+1.9}{x_{4}}-1\leq 0,\\ g_{11}\left(\overset{⟶}{x}\right)=\frac{1.1x_{7}+1.9}{x_{5}}-1\leq 0. \end{array}$$

Variable range

(39) $$\begin{array}{c} 2.6\leq x_{1}\leq 3.6,\\ 0.7\leq x_{2}\leq 0.8,\\ 17\leq x_{3}\leq 28,\\ 7.3\leq x_{4}\leq 8.3,\\ 7.8\leq x_{5}\leq 8.3,\\ 2.9\leq x_{6}\leq 3.9,\\ 5.0\leq x_{7}\leq 5.5. \end{array}$$

Table 13 shows the test results that demonstrate the proposed algorithm's effectiveness in obtaining the optimal values for solving this problem.

## 5. Conclusion

In this paper, an improved HHO algorithm named ERHHO is proposed to overcome the shortcoming of the basic HHO algorithm. The ERHHO algorithm starts with initializing population positions, where we introduced the tent chaotic map to improve the diversity. And then three phases: exploration, transaction from exploration to exploitation, and exploitation, are performed. We proposed an exploration factor to update the formula to expand the global search range at the exploration phase. And, at the phase of exploitation, we proposed a random walk strategy after four hunting strategies to effectively improve the ability to find more accurate results. Twenty-three standard benchmark functions evaluate the proposed algorithm's ability in the stage of exploration and exploitation. The results verified that the proposed ERHHO algorithm can yield very effective outcomes and get almost the best results compared to the other algorithms. Then the Wilcoxon signed-rank test is used to demonstrate the significant differences between ERHHO and other competing algorithms. The algorithm's superiority is further demonstrated by testing on five engineering design problems and CEC2017 test functions for real problems. Furthermore, some challenges in the real world can be solved by using ERHHO properly, such as feature selection, multithreshold image segmentation, convolution neural network, and so on. For further verification, another inquiry will be performed on whether this hybrid method can improve the performance of other optimization algorithms.

## Figures and Tables

**Figure 1:** Different phases of HHO [36].

**Figure 2:** Ten commonly used chaotic maps.

**Figure 3:** Cos function convergence curve.

**Figure 4:** Curve of exploration factor.

**Figure 5:** Flowchart of ERHHO.

**Figure 6:** Convergence curves of 23 benchmark functions: (a) F3, (b) F5, (c) F7, (d) F8, (e) F9, (f) F10, (g) F12, (h) F13, (i) F14, (j) F15, (k) F19, (l) F20, (m) F21, (n) F22, and (o) F23.

**Figure 7:** Friedman mean ranking for each type of CEC2017 test functions.

**Figure 8:** Tension spring design problem [50].

**Figure 9:** Pressure vessel design problem [50].

**Figure 10:** Three-bar truss design problem [50].

**Figure 11:** Cantilever beam design [55].

**Figure 12:** Speed reducer problem [55].

**Algorithm 1:** Pseudocode of ERHHO.

**Table 1:** Benchmark function properties (Dim indicates dimension).

Function		Dim	Range	*F*_min_
Unimodal benchmark functions	F1	30	[−100, 100]	0
	F2	30	[−10, 10]	0
	F3	30	[−100, 100]	0
	F4	30	[−100, 100]	0
	F5	30	[−30, 30]	0
	F6	30	[−100, 100]	0
	F7	30	[−1.28, 1.28]	0

Multimodal benchmark functions	F8	30	[−500, 500]	418.9829 × dim
	F9	30	[−5.12, 5.12]	
	F10	30	[−32, 32]	0
	F11	30	[−600, 600]	0
	F12	30	[−50, 50]	0
	F13	30	[−50, 50]	0

Fixed-dimension multimodal benchmark functions	F14	2	[−65, 65]	0.998
	F15	4	[−5, 5]	0.00030
	F16	2	[−5, 5]	−1.0316
	F17	2	[−5, 5]	0.398
	F18	2	[−2, 2]	3
	F19	3	[−1, 2]	−3.86
	F20	6	[0, 1]	−3.32
	F21	4	[0, 10]	−10.1532
	F22	4	[0, 10]	−10.4028
	F23	4	[0, 10]	−10.5363

**Table 2:** Parameter settings for the comparative algorithms.

Algorithm	Parameters
ERHHO	*β* = 1.5, *a* = 0.7, *b* = 2, *c* = 6
SMA [27]	*z* = 0.03
WOA [24]	*a*_1_ = [2, 0], *a*_2_ = [−2, 1], *b* = 1
SSA [25]	*c*_1_ ∈ [0, 1], *c*_2_ ∈ [0, 1]
SCA [26]	*a* = 2
HHO [36]	*β* = 1.5
DHHO/M [43]	*a* = 2.5, *F* = 0.5
HHOCM [41]	*β* = 1.5

**Table 3:** Parameters sensitivity analysis.

Function	*b* = 2	*b* = 2	*b* = 2	*b* = 4	*b* = 4	*b* = 4	*b* = 6	*b* = 6	*b* = 6
	*c* = 2	*c* = 4	*c* = 6	*c* = 2	*c* = 4	*c* = 6	*c* = 2	*c* = 4	*c* = 6
F1	**0.0000E + 00**	**0.0000E + 00**	**0.0000E + 00**	**0.0000E + 00**	**0.0000E + 00**	**0.0000E + 00**	**0.0000E + 00**	**0.0000E + 00**	**0.0000E + 00**
F2	**0.0000E + 00**	**0.0000E + 00**	**0.0000E + 00**	**0.0000E + 00**	**0.0000E + 00**	**0.0000E + 00**	**0.0000E + 00**	**0.0000E + 00**	**0.0000E + 00**
F3	**0.0000E + 00**	**0.0000E + 00**	**0.0000E + 00**	**0.0000E + 00**	**0.0000E + 00**	**0.0000E + 00**	**0.0000E + 00**	**0.0000E + 00**	**0.0000E + 00**
F4	**0.0000E + 00**	**0.0000E + 00**	**0.0000E + 00**	**0.0000E + 00**	**0.0000E + 00**	**0.0000E + 00**	**0.0000E + 00**	**0.0000E + 00**	**0.0000E + 00**
F5	4.1086*E* − 04	2.3293*E* − 04	**9.9757E − 05**	4.4925*E* − 04	2.4795*E* − 04	1.6512*E* − 04	1.5639*E* − 03	3.3876*E* − 04	4.1522*E* − 04
F6	9.1737*E* − 05	3.8910*E* − 05	**1.4826E − 05**	8.5754*E* − 05	5.2338*E* − 05	4.6220*E* − 05	1.7327*E* − 04	1.1701*E* − 04	3.8893*E* − 05
F7	**5.7338E − 05**	8.4463*E* − 05	7.1416*E* − 05	6.3548*E* − 05	7.9739*E* − 05	7.3938*E* − 05	7.3475*E* − 05	6.7715*E* − 05	6.3104*E* − 05
F8	**−1.2569E + 04**	**−1.2569E + 04**	**−1.2569E + 04**	**−1.2569E + 04**	**−1.2569E + 04**	**−1.2569E + 04**	**−1.2569E + 04**	**−1.2569E + 04**	**−1.2569E + 04**
F9	**0.0000E + 00**	**0.0000E + 00**	**0.0000E + 00**	**0.0000E + 00**	**0.0000E + 00**	**0.0000E + 00**	**0.0000E + 00**	**0.0000E + 00**	**0.0000E + 00**
F10	**8.8818E − 16**	**8.8818E − 16**	**8.8818E − 16**	**8.8818E − 16**	**8.8818E − 16**	**8.8818E − 16**	**8.8818E − 16**	**8.8818E − 16**	**8.8818E − 16**
F11	**0.0000E + 00**	**0.0000E + 00**	**0.0000E + 00**	**0.0000E + 00**	**0.0000E + 00**	**0.0000E + 00**	**0.0000E + 00**	**0.0000E + 00**	**0.0000E + 00**
F12	1.9085*E* − 06	6.3102*E* − 07	**2.9078E − 07**	4.8068*E* − 06	1.8862*E* − 06	1.8322*E* − 06	6.5051*E* − 06	2.0196*E* − 06	2.2776*E* − 06
F13	2.6364*E* − 05	8.3301*E* − 06	**4.8525E − 06**	5.0282*E* − 05	1.7997*E* − 05	1.8399*E* − 05	4.8097*E* − 05	4.7190*E* − 05	2.8779*E* − 05
F14	**9.9800E − 01**	**9.9800E − 01**	**9.9800E − 01**	**9.9800E − 01**	1.1303*E* + 00	1.0311*E* + 00	**9.9800E − 01**	1.3599*E* + 00	**9.9800E − 01**
F15	3.2234*E* − 04	3.4356*E* − 04	3.3924*E* − 04	3.6062*E* − 04	3.4211*E* − 04	**3.0770E − 04**	3.2145*E* − 04	3.1080*E* − 04	3.6977*E* − 04
F16	**−1.0316E + 00**	**−1.0316E + 00**	**−1.0316E + 00**	**−1.0316E + 00**	**−1.0316E + 00**	**−1.0316E + 00**	**−1.0316E + 00**	**−1.0316E + 00**	**−1.0316E + 00**
F17	**3.9789E − 01**	**3.9789E − 01**	**3.9789E − 01**	**3.9789E − 01**	**3.9789E − 01**	**3.9789E − 01**	**3.9789E − 01**	**3.9789E − 01**	**3.9789E − 01**
F18	**3.0000E + 00**	**3.0000E + 00**	**3.0000E + 00**	**3.0000E + 00**	**3.0000E + 00**	**3.0000E + 00**	**3.0000E + 00**	**3.0000E + 00**	**3.0000E + 00**
F19	**−3.8628E + 00**	**−3.8628E + 00**	**−3.8628E + 00**	**−3.8628E + 00**	**−3.8628E + 00**	**−3.8628E + 00**	**−3.8628E + 00**	**−3.8628E + 00**	**−3.8628E + 00**
F20	−3.2268*E* + 00	−3.2558*E* + 00	−3.2689*E* + 00	−3.1938*E* + 00	−3.2562*E* + 00	−3.2735*E* + 00	−3.2015*E* + 00	**−3.2816E + 00**	−3.2741*E* + 00
F21	−1.0152*E* + 01	**−1.0153E + 01**	**−1.0153E + 01**	−1.0152*E* + 01	**−1.0153E + 01**	**−1.0153E + 01**	**−1.0153E + 01**	**−1.0153E + 01**	**−1.0153E + 01**
F22	−1.0402*E* + 01	**−1.0403E + 01**	**−1.0403E + 01**	−1.0402*E* + 01	**−1.0403E + 01**	**−1.0403E + 01**	−1.0402*E* + 01	**−1.0403E + 01**	**−1.0403E + 01**
F23	−1.0536*E* + 01	**−1.0536E + 01**	**−1.0536E + 01**	−1.0536*E* + 01	**−1.0536E + 01**	**−1.0536E + 01**	−1.0535*E* + 01	**−1.0536E + 01**	**−1.0536E + 01**
Sum	14	16	**20**	13	14	16	14	16	16

The best results are marked in bold.

**Table 4:** Results of algorithms on 23 benchmark functions.

Function		ERHHO	SMA	WOA	SSA	SCA	HHO	DHHO/M	HHOCM
F1	Mean	**0.0000E + 00**	5.4841*e* − 322	7.8586*E* − 74	4.5572*E* − 07	1.5650*E* + 01	2.4246*E* − 96	1.9672*E* − 95	**0.0000E + 00**
	Std	**0.0000E + 00**	**0.0000E + 00**	2.1680*E* − 73	8.0901*E* − 07	2.1910*E* + 01	1.3093*E* − 95	6.7432*E* − 95	**0.0000E + 00**

F2	Mean	**0.0000E + 00**	1.9735*E* − 150	4.7683*E* − 51	2.4203*E* + 00	2.4894*E* − 02	2.9318*E* − 51	1.3176*E* − 48	1.2225*E* − 203
	Std	**0.0000E + 00**	1.0809*E* − 149	2.0969*E* − 50	1.7085*E* + 00	3.5592*E* − 02	1.1152*E* − 50	6.0671*E* − 48	**0.0000E + 00**

F3	Mean	**0.0000E + 00**	2.0792*E* − 281	4.4988*E* + 04	1.4407*E* + 03	9.3775*E* + 03	8.4362*E* − 73	7.6735*E* − 70	**0.0000E + 00**
	Std	**0.0000E + 00**	**0.0000E + 00**	1.2599*E* + 04	9.7094*E* + 02	5.8048*E* + 03	4.6060*E* − 72	4.2027*E* − 69	**0.0000E + 00**

F4	Mean	**0.0000E + 00**	2.1129*E* − 137	3.8143*E* + 01	1.1509*E* + 01	3.2926*E* + 01	5.4154*E* − 49	3.9550*E* − 43	4.5525*E* − 197
	Std	**0.0000E + 00**	1.1573*E* − 136	2.7276*E* + 01	3.7852*E* + 00	1.3070*E* + 01	1.4703*E* − 48	2.1642*E* − 42	**0.0000E + 00**

F5	Mean	**8.9883E − 05**	8.3666*E* + 00	2.7925*E* + 01	2.7609*E* + 02	4.3940*E* + 04	1.0142*E* − 02	6.7040*E* − 03	3.1438*E* − 02
	Std	**1.9452E − 04**	1.1685*E* + 01	4.5946*E *** − **01	3.6619*E* + 02	6.4024*E* + 04	1.2554*E* − 02	9.5798*E* − 03	5.0191*E* − 02

F6	Mean	1.6455*E* − 05	5.2944*E* − 03	4.4446*E* − 01	**2.0747E − 07**	1.9795*E* + 01	1.5127*E* − 04	7.3876*E* − 05	3.1254*E* − 04
	Std	2.5216*E* − 05	4.1571*E* − 03	2.8101*E* − 01	**4.6645E − 07**	1.8292*E* + 01	1.7402*E* − 04	1.0886*E* − 04	3.8262*E* − 04

F7	Mean	**7.6595E − 05**	2.1094*E* − 04	2.0569*E* − 03	1.6531*E* − 01	9.7607*E* − 02	1.3707*E* − 04	1.5754*E* − 04	1.6184*E* − 04
	Std	**5.8914E − 05**	1.7724*E* − 04	2.0834*E* − 03	7.4193*E* − 02	7.9845*E* − 02	1.0626*E* − 04	1.4448*E* − 04	1.7591*E* − 04

F8	Mean	**−1.2569E + 04**	**−1.2569E + 04**	−1.0181*E* + 04	−7.4877*E* + 03	−3.8109*E* + 03	**−1.2569E + 04**	−1.2469*E* + 04	−1.2554*E* + 04
	Std	**5.0470E − 02**	3.5003*E* − 01	1.6535*E* + 03	6.3231*E* + 02	3.4249*E* + 02	8.9555*E* − 01	5.4333*E* + 02	5.4994*E* + 01

F9	Mean	**0.0000E + 00**	**0.0000E + 00**	3.7896*E*−15	4.9483*E* + 01	4.6372*E* + 01	**0.0000E + 00**	**0.0000E + 00**	**0.0000E + 00**
	Std	**0.0000E + 00**	**0.0000E + 00**	2.0756*E*−14	1.3277*E* + 01	3.4053*E* + 01	**0.0000E + 00**	**0.0000E + 00**	**0.0000E + 00**

F10	Mean	**8.8818E − 16**	**8.8818E − 16**	5.3883*E* − 15	2.7147*E* + 00	1.2192*E* + 01	**8.8818E − 16**	**8.8818E − 16**	**8.8818E − 16**
	Std	**0.0000E + 00**	**0.0000E + 00**	2.0723*E* − 15	9.8679*E* − 01	9.4808*E* + 00	**0.0000E + 00**	**0.0000E + 00**	**0.0000E + 00**

F11	Mean	**0.0000E + 00**	**0.0000E + 00**	1.6696*E* − 02	1.7711*E* − 02	9.7236*E* − 01	**0.0000E + 00**	**0.0000E + 00**	**0.0000E + 00**
	Std	**0.0000E + 00**	**0.0000E + 00**	5.4084*E* − 02	1.4171*E* − 02	3.5476*E* − 01	**0.0000E + 00**	**0.0000E + 00**	**0.0000E + 00**

F12	Mean	**3.1435E − 07**	4.9064*E* − 03	2.1150*E* − 02	6.6186*E* + 00	2.4854*E* + 04	1.3945*E* − 05	8.5284*E* − 06	1.5684*E* − 05
	Std	**5.0819E − 07**	5.8190*E* − 03	1.3549*E* − 02	2.8000*E* + 00	8.6251*E* + 04	2.0991*E* − 05	1.0043*E* − 05	2.2746*E* − 05

F13	Mean	**7.2242E − 06**	7.2277*E* − 03	5.0105*E* − 01	1.1788*E* + 01	1.1416*E* + 05	7.4801*E* − 05	9.5150*E* − 05	2.7612*E* − 04
	Std	**9.7389E − 06**	6.6267*E* − 03	1.8495*E* − 01	1.2856*E* + 01	2.8677*E* + 05	8.4403*E* − 05	1.0966*E* − 04	3.9597*E* − 04

F14	Mean	**9.9800E − 01**	**9.9800E − 01**	2.7353*E* + 00	1.1637*E* + 00	1.7223*E* + 00	1.7549*E* + 00	1.2949*E* + 00	1.1634*E* + 00
	Std	7.4084*E* − 11	**5.6156E − 13**	2.8639*E* + 00	3.7678*E*−01	1.8868*E* + 00	1.6921*E* + 00	9.3994*E* − 01	5.2656*E* − 01

F15	Mean	**3.1210E − 04**	5.6703*E* − 04	6.9856*E* − 04	2.1817*E* − 03	1.0610*E* − 03	3.8687*E* − 04	4.5821*E* − 04	5.6125*E* − 04
	Std	**2.1452E − 05**	3.0981*E* − 04	4.7771*E* − 04	4.9506*E* − 03	4.1995*E* − 04	2.8444*E* − 04	3.0067*E* − 04	4.2913*E* − 04

F16	Mean	**−1.0316E + 00**	**−1.0316E + 00**	**−1.0316E + 00**	**1.0316E + 00**	**−1.0316E + 00**	**−1.0316E + 00**	**−1.0316E + 00**	**−1.0316E + 00**
	Std	**4.8085E − 16**	2.4615*E* − 09	1.2442*E* − 09	3.3423*E* − 14	5.2063*E* − 05	4.2516*E* − 09	5.7528*E* − 11	3.8734*E* − 09

F17	Mean	**3.9789E − 01**	**3.9789E − 01**	**3.9789E − 01**	**3.9789E − 01**	3.9998*E*−01	**3.9789E − 01**	**3.9789E − 01**	**3.9789E − 01**
	Std	**1.1571E − 15**	2.0433*E *** **−** **07	8.4094*E *** **−** **06	1.8281*E *** **−** **14	2.1427*E *** **−** **03	7.6834*E *** **−** **06	3.9921*E *** **−** **06	1.6521*E *** **−** **06

F18	Mean	**3.0000E + 00**	**3.0000E + 00**	**3.0000E + 00**	**3.0000E + 00**	3.0001*E* + 00	**3.0000E + 00**	**3.0000E + 00**	**3.0000E + 00**
	Std	**1.1106E − 14**	1.8331*E *** **−** **10	3.8495*E *** **−** **05	3.0811*E *** **−** **13	1.3607*E *** **−** **04	3.3143*E *** **−** **07	7.5272*E *** **−** **08	1.5483*E *** **−** **08

F19	Mean	−3.8628*E* + 00	−3.8628*E* + 00	−3.8532*E* + 00	−3.8628*E* + 00	−3.8543*E* + 00	−3.8599*E* + 00	**−3.8608E + 00**	−3.8626*E* + 00
	Std	**8.0972E − 15**	3.3188*E*−07	1.1608*E*−02	7.2861*E*−11	2.5528*E*−03	4.2515*E*−03	3.0862*E*−03	5.1550*E*−04

F20	Mean	**−3.2692E + 00**	−3.2621*E* + 00	−3.2474*E* + 00	−3.2178*E* + 00	−2.9363*E* + 00	−3.0985*E* + 00	−3.1112*E* + 00	−3.2615*E* + 00
	Std	6.1618*E *** **−** **02	6.0867*E *** **−** **02	9.7561*E *** **−** **02	**4.7860E−02**	2.6267*E *** **−** **01	1.1844*E *** **−** **01	8.3931*E *** **−** **02	6.7841*E *** **−** **02
F21	Mean	**−1.0153E + 01**	**−1.0153E + 01**	−8.7154*E* + 00	−7.0613*E* + 00	−2.1979*E* + 00	−5.0516*E* + 00	−1.0032*E* + 01	−5.0550*E* + 00
	Std	**3.0528E − 05**	3.2280*E *** **−** **04	2.2751*E* + 00	3.4592*E* + 00	1.7374*E* + 00	3.1444*E *** **−** **03	1.2614*E *** **−** **01	2.6879*E *** **−** **04

F22	Mean	**−1.0403E + 01**	**−1.0403E + 01**	−8.8619*E* + 00	−8.4885*E* + 00	−2.7876*E* + 00	−5.0047*E* + 00	−1.0212*E* + 01	−5.0876*E* + 00
	Std	**1.1586E − 07**	2.0872*E *** **−** **04	2.6262*E* + 00	3.0306*E* + 00	1.7662*E* + 00	4.2878*E *** **−** **01	1.8693*E *** **−** **01	1.0644*E *** **−** **04

F23	Mean	**−1.0536E + 01**	**−1.0536E + 01**	−7.8012*E* + 00	−8.6030*E* + 00	−4.2432*E* + 00	−5.4760*E* + 00	−1.0404*E* + 01	−5.1283*E* + 00
	Std	**4.5569E−07**	3.6654*E *** **−** **04	3.0292*E* + 00	3.0771*E* + 00	1.7263*E* + 00	1.3367*E* + 00	1.5417*E *** **−** **01	1.7786*E *** **−** **04

The best results are marked as bold fonts. For the unimodal benchmark functions (F1–F7), ERHHO can obtain the best result except for F6.

**Table 5:** Results of HHO (hybrid exploration factor) on F21–F23.

Function		HHO	HHO + exploration factor
F21	Mean	−5.3410*E* + 00	**−1.0147E + 01**
	Std	1.1097*E* + 00	**7.5648E − 03**

F22	Mean	−5.2560*E* + 00	**−1.0394E + 01**
	Std	9.5700*E* − 01	**1.4686E − 02**

F23	Mean	−5.3039*E* + 00	**−1.0530E + 01**
	Std	9.8154*E* − 01	**6.1909E − 03**

The best results are marked in bold.

**Table 6:** The results of the Wilcoxon signed test.

Function	ERHHO vs.						
	SMA	WOA	SSA	SCA	HHO	DHHO/M	HHOCM
F1	**NaN**	6.8662*E* − 07	6.8662*E* − 07	6.8662*E* − 07	6.8662*E* − 07	6.8662*E* − 07	**NaN**
F2	6.8662*E* − 07	6.8662*E* − 07	6.8662*E* − 07	6.8662*E* − 07	6.8662*E* − 07	6.8662*E* − 07	6.8662*E* − 07
F3	**7.9725E − 02**	6.8662*E* − 07	6.8662*E* − 07	6.8662*E* − 07	6.8662*E* − 07	6.8662*E* − 07	**NaN**
F4	6.8662*E* − 07	6.8662*E* − 07	6.8662*E* − 07	6.8662*E* − 07	6.8662*E* − 07	6.8662*E* − 07	6.8662*E* − 07
F5	4.1432*E* − 06	3.3918*E* − 06	3.3918*E* − 06	3.3918*E* − 06	3.6093*E* − 04	3.3568*E* − 05	7.4772*E* − 06
F6	3.3918*E* − 06	3.3918*E* − 06	3.3918*E* − 06	3.3918*E* − 06	**5.3383E − 01**	**1.5846E − 01**	7.9403*E* − 03
F7	4.2111*E* − 02	3.3918*E* − 06	3.3918*E* − 06	3.3918*E* − 06	**1.0574E − 01**	1.4397*E* − 02	6.1898*E* − 03
F8	1.9352*E* − 05	3.3918*E* − 06	3.3918*E* − 06	3.3918*E* − 06	9.6615*E* − 05	1.1457*E* − 04	5.4521*E* − 03
F9	**NaN**	**3.5065E − 01**	6.8662*E* − 07	6.8662*E* − 07	**NaN**	**NaN**	**NaN**
F10	**NaN**	2.1523*E* − 05	6.8662*E* − 07	6.8662*E* − 07	**NaN**	**NaN**	**NaN**
F11	**NaN**	**3.5065E − 01**	6.8662*E* − 07	6.8662*E* − 07	**NaN**	**NaN**	**NaN**
F12	3.3918*E* − 06	3.3918*E* − 06	3.3918*E* − 06	3.3918*E* − 06	7.0162*E* − 03	4.2111*E* − 02	2.8226*E* − 03
F13	3.3918*E* − 06	3.3918*E* − 06	3.3918*E* − 06	3.3918*E* − 06	1.0992*E* − 05	1.0500*E* − 03	2.2289*E* − 04
F14	5.2468*E* − 03	3.0947*E* − 05	**2.7876E − 01**	3.0659*E* − 06	6.3415*E* − 05	5.3134*E* − 05	3.5402*E* − 03
F15	3.3918*E* − 06	4.1432*E* − 06	5.0527*E* − 06	3.3918*E* − 06	1.0992*E* − 05	1.1457*E* − 04	4.0200*E* − 05
F16	1.2604*E* − 06	1.2604*E* − 06	1.2604*E* − 06	1.2604*E* − 06	1.2604*E* − 06	1.5660*E* − 06	1.2604*E* − 06
F17	2.2038*E* − 06	2.2038*E* − 06	3.4080*E* − 04	2.2038*E* − 06	4.9642*E* − 06	1.9074*E* − 05	2.4387*E* − 06
F18	5.0162*E* − 06	3.3664*E* − 06	1.0918*E* − 05	3.3664*E* − 06	3.3664*E* − 06	3.9725*E* − 05	3.3664*E* − 06
F19	3.2092*E* − 06	3.2092*E* − 06	5.5823*E* − 04	3.2092*E* − 06	3.2092*E* − 06	3.2092*E* − 06	3.2092*E* − 06
F20	**2.4549E − 01**	**5.6145E − 01**	1.0122*E* − 02	3.3918*E* − 06	4.7948*E* − 03	2.4626*E* − 03	**8.6823E − 01**
F21	1.6053*E* − 05	3.3918*E* − 06	**7.7155E − 01**	3.3918*E* − 06	3.3918*E* − 06	3.3918*E* − 06	3.3918*E* − 06
F22	7.4772*E* − 06	3.3918*E* − 06	**1.2486E − 01**	3.3918*E* − 06	3.3918*E* − 06	3.3918*E* − 06	3.3918*E* − 06
F23	4.8063*E* − 05	3.3918*E* − 06	5.7371*E* − 05	3.3918*E* − 06	3.3918*E* − 06	4.1432*E* − 06	3.3918*E* − 06
(W|L|T)	(17|2|4)	(20|3|0)	(20|3|0)	(23|0|0)	(18|2|3)	(19|1|3)	(17|1|5)

The best results are marked in bold.

**Table 7:** Properties and summary of the CEC2017.

Type	No.	Functions	Global min	Domain
Unimodal function	F1	Shifted and rotated bent cigar function	100	[−100, 100]
	F2	Shifted and rotated sum of different power function	200	[−100, 100]
	F3	Shifted and rotated Zakharov's function	300	[−100, 100]

Multimodal functions	F4	Shifted and rotated Rosenbrock's function	400	[−100, 100]
	F5	Shifted and rotated Rastrigin's function	500	[−100, 100]
	F6	Shifted and rotated expanded Schaffer's function	600	[−100, 100]
	F7	Shifted and rotated Lunacek Bi_Rastrigin function	700	[−100, 100]
	F8	Shifted and rotated noncontinuous Rastrigin's function	800	[−100, 100]
	F9	Shifted and rotated Levy function	900	[−100, 100]
	F10	Shifted and rotated Schwefel's function	1,000	[−100, 100]

Hybrid functions	F11	Hybrid function of Zakharov, Rosenbrock, and Rastrigin	1,100	[−100, 100]
	F12	Hybrid function of high conditioned elliptic, modified Schwefel, and bent cigar	1,200	[−100, 100]
	F13	Hybrid function of bent cigar, Rosenbrock, and Lunacek bi-Rastrigin	1,300	[−100, 100]
	F14	Hybrid function of elliptic, Ackley, Schaffer and Rastrigin	1,400	[−100, 100]
	F15	Hybrid function of bent cigar, HGBat, Rastrigin, and Rosenbrock	1,500	[−100, 100]
	F16	Hybrid function of expanded Schaffer, HGBat, Rosenbrock, and modified Schwefel	1,600	[−100, 100]
	F17	Hybrid function of Katsuura, Ackley, expanded Griewank plus Rosenbrock, modified Schwefel, and Rastrigin	1,700	[−100, 100]
	F18	Hybrid function of high conditioned elliptic, Ackley, Rastrigin, HGBat, and Discus	1,800	[−100, 100]
	F19	Hybrid function of bent cigar, Rastrigin, expanded Griewank plus Rosenbrock, Weierstrass, and expanded Schaffer	1,900	[−100, 100]
	F20	Hybrid function of HappyCat, Katsuura, Ackley, Rastrigin, modified Schwefel, and Schaffer	2,000	[−100, 100]

Composition functions	F21	Composition function of Rosenbrock, high conditioned elliptic, and Rastrigin	2,100	[−100, 100]
	F22	Composition function of Rastrigin's, Griewank, and modified Schwefel	2,200	[−100, 100]
	F23	Composition function of Rosenbrock, Ackley, modified Schwefel, and Rastrigin	2,300	[−100, 100]
	F24	Composition function of Ackley, high conditioned elliptic, Griewank, and Rastrigin	2,400	[−100, 100]
	F25	Composition function of Rastrigin, HappyCat, Ackley, Discus, and Rosenbrock	2,500	[−100, 100]
	F26	Composition function of expanded Schaffer, modified Schwefel, Griewank, Rosenbrock, and Rastrigin	2,600	[−100, 100]
	F27	Composition function of HGBat, Rastrigin, modified Schwefel, bent cigar, high conditioned elliptic, and expanded Schaffer	2,700	[−100, 100]
	F28	Composition function of Ackley, Griewank, Discus, Rosenbrock, HappyCat, and expanded Schaffer	2,800	[−100, 100]
	F29	Composition function of shifted and rotated Rastrigin, expanded Schaffer, and Lunacek Bi_Rastrigin	2,900	[−100, 100]
	F30	F30 composition function of shifted and rotated Rastrigin, noncontinuous Rastrigin, and Levy function	3,000	[−100, 100]

**Table 8:** The results of CEC2017 test functions.

Type	No.		ERHHO	HHO	DHHO/M	HHOCM	CEHHO
Unimodal function	F1	Mean	**1.2052E + 04**	3.6019*E* + 05	4.2939*E* + 05	2.0170*E* + 04	1.0067*E* + 06
		Std	**2.2216E + 04**	1.7863*E* + 05	3.0607*E* + 05	2.4823*E* + 04	1.0026*E* + 06
		Rank	**1**	3	4	2	5
	F3	Mean	3.0063*E* + 02	3.0180*E* + 02	3.0231*E* + 02	**3.0019E + 02**	3.1873*E* + 02
		Std	4.6904*E* − 01	1.0312*E* + 00	2.0173*E* + 00	**9.7727E − 02**	1.6569*E* + 01
		Rank	2	3	4	**1**	5

Multimodal functions	F4	Mean	4.1270*E* + 02	4.1578*E* + 02	4.1392*E* + 02	**4.0689E + 02**	4.1280*E* + 02
		Std	2.1283*E* + 01	2.5703*E* + 01	2.1889*E* + 01	**1.1731E + 01**	1.9551*E* + 01
		Rank	2	5	4	**1**	3
	F5	Mean	**5.4272E + 02**	5.4457*E* + 02	5.4797*E* + 02	5.4413*E* + 02	5.4567*E* + 02
		Std	**1.7715E + 01**	1.2083*E* + 01	1.3398*E* + 01	1.5229*E* + 01	1.8236*E* + 01
		Rank	**1**	3	5	2	4
	F6	Mean	**6.2997E + 02**	6.3151*E* + 02	6.3265*E* + 02	6.3046*E* + 02	6.3753*E* + 02
		Std	**9.6724E + 00**	1.2635*E* + 01	1.1154*E* + 01	1.0670*E* + 01	1.2120*E* + 01
		Rank	**1**	3	4	2	5
	F7	Mean	7.8617*E* + 02	7.8076*E* + 02	7.7761*E* + 02	**7.7481E + 02**	7.8152*E* + 02
		Std	1.8646*E* + 01	1.6252*E* + 01	1.7448*E* + 01	**2.0940E + 01**	2.2054*E* + 01
		Rank	5	3	2	**1**	4
	F8	Mean	8.3287*E* + 02	8.2779*E* + 02	8.2843*E* + 02	8.2989*E* + 02	**8.2428E + 02**
		Std	6.4227*E* + 00	8.0354*E* + 00	7.6805*E* + 00	8.9310*E* + 00	**7.6576E + 00**
		Rank	5	2	3	4	**1**
	F9	Mean	1.3612*E* + 03	1.4738*E* + 03	1.3986*E* + 03	1.4321*E* + 03	**1.3168E + 03**
		Std	3.0596*E* + 02	2.0219*E* + 02	2.0034*E* + 02	2.5386*E* + 02	**1.9220E + 02**
		Rank	2	5	3	4	**1**
	F10	Mean	**1.9272E + 03**	1.9801*E* + 03	2.0096*E* + 03	2.0094*E* + 03	2.0899*E* + 03
		Std	**2.6782E + 02**	3.0179*E* + 02	2.8965*E* + 02	2.9359*E* + 02	3.1406*E* + 02
		Rank	**1**	2	4	3	5

Hybrid functions	F11	Mean	**1.1567E + 03**	1.1797*E* + 03	1.1939*E* + 03	1.1647*E* + 03	1.1809*E* + 03
		Std	**4.3639E + 01**	8.0529*E* + 01	9.0864*E* + 01	5.1621*E* + 01	6.2806*E* + 01
		Rank	**1**	3	5	2	4
	F12	Mean	**2.5268E + 04**	2.3910*E* + 06	2.6341*E* + 06	2.5694*E* + 06	2.8299*E* + 06
		Std	**3.7776E + 04**	2.0613*E* + 06	2.9949*E* + 06	2.8868*E* + 06	3.1678*E* + 06
		Rank	**1**	2	4	3	5
	F13	Mean	**2.6880E + 03**	1.7767*E* + 04	2.0431*E* + 04	1.2350*E* + 04	1.4179*E* + 04
		Std	**2.2783E + 03**	1.1560*E* + 04	1.1932*E* + 04	9.9645*E* + 03	8.7188*E* + 03
		Rank	**1**	4	5	2	3
	F14	Mean	**1.4865E + 03**	1.5791*E* + 03	1.5321*E* + 03	1.5857*E* + 03	1.5634*E* + 03
		Std	**2.4693E + 01**	2.0948*E* + 02	3.4605*E* + 01	1.9928*E* + 02	8.5603*E* + 01
		Rank	**1**	4	2	5	3
	F15	Mean	**1.5942E + 03**	4.0799*E* + 03	4.2891*E* + 03	4.6614*E* + 03	6.3234*E* + 03
		Std	**5.7397E + 01**	1.7066*E* + 03	2.0041*E* + 03	1.7606*E* + 03	2.8184*E* + 03
		Rank	**1**	2	3	4	5
	F16	Mean	1.9278*E* + 03	1.8955*E* + 03	**1.8830E + 03**	1.9312*E* + 03	1.8949*E* + 03
		Std	1.2443*E* + 02	1.5078*E* + 02	**1.3381E + 02**	1.5608*E* + 02	1.4804*E* + 02
		Rank	4	3	**1**	5	2
	F17	Mean	1.7674*E* + 03	1.7769*E* + 03	1.7841*E* + 03	**1.7664E + 03**	1.7967*E* + 03
		Std	2.4383*E* + 01	2.8229*E* + 01	6.0168*E* + 01	**2.1723E + 01**	3.8642*E* + 01
		Rank	2	3	4	**1**	5
	F18	Mean	**3.8251E + 03**	1.3844*E* + 04	1.6139*E* + 04	1.7430*E* + 04	1.5003*E* + 04
		Std	**3.7128E + 03**	1.1177*E* + 04	1.1613*E* + 04	1.0382*E* + 04	1.2422*E* + 04
		Rank	**1**	2	4	5	3
	F19	Mean	**4.7207E + 03**	1.1593*E* + 04	1.2784*E* + 04	1.2917*E* + 04	1.5813*E* + 04
		Std	**5.0189E + 03**	1.1274*E* + 04	1.1131*E* + 04	1.1182*E* + 04	1.3094*E* + 04
		Rank	**1**	2	3	4	5
	F20	Mean	**2.1509E + 03**	2.1761*E* + 03	2.1553*E* + 03	2.1520*E* + 03	2.1662*E* + 03
		Std	**6.1600E + 01**	6.3993*E* + 01	6.5874*E* + 01	7.4938*E* + 01	6.8566*E* + 01
		Rank	**1**	5	3	2	4

Composition functions	F21	Mean	2.3271*E* + 03	2.3298*E* + 03	2.3117*E* + 03	2.3291*E* + 03	**2.3016E + 03**
		Std	5.1674*E* + 01	5.1905*E* + 01	6.1347*E* + 01	6.0511*E* + 01	**6.3126E + 01**
		Rank	3	5	2	4	**1**
	F22	Mean	**2.3123E + 03**	2.3776*E* + 03	2.3159*E* + 03	2.3580*E* + 03	2.3759*E* + 03
		Std	**6.4041E + 00**	3.4445*E* + 02	6.1462*E* + 00	2.7117*E* + 02	2.4397*E* + 02
		Rank	**1**	5	2	3	4
	F23	Mean	2.6610*E* + 03	2.6651*E* + 03	**2.6565E + 03**	2.6833*E* + 03	2.6664*E* + 03
		Std	2.3793*E* + 01	2.7693*E* + 01	**2.6149E + 01**	2.5521*E* + 01	3.0349*E* + 01
		Rank	2	3	**1**	5	4
	F24	Mean	2.7871*E* + 03	2.7876*E* + 03	2.7977*E* + 03	2.8124*E* + 03	**2.7837E + 03**
		Std	9.6226*E* + 01	1.0482*E* + 02	7.3836*E* + 01	9.2546*E* + 01	**8.1668E + 01**
		Rank	2	3	4	5	**1**
	F25	Mean	**2.9141E + 03**	2.9389*E* + 03	2.9331*E* + 03	2.9168*E* + 03	2.9448*E* + 03
		Std	**6.4027E + 01**	3.7666*E* + 01	2.4771*E* + 01	8.8852*E* + 01	3.4255*E* + 01
		Rank	**1**	4	3	2	5
	F26	Mean	3.4378*E* + 03	**3.3932E + 03**	3.4342*E* + 03	3.4730*E* + 03	3.7968*E* + 03
		Std	6.6555*E* + 02	**5.4030E + 02**	5.9523*E* + 02	4.9775*E* + 02	5.8494*E* + 02
		Rank	3	**1**	2	4	5
	F27	Mean	**3.1341E + 03**	3.1412*E* + 03	3.1451*E* + 03	3.1499*E* + 03	3.1616*E* + 03
		Std	**3.8294E + 01**	4.5307*E* + 01	4.3369*E* + 01	3.2091*E* + 01	4.6269*E* + 01
		Rank	**1**	2	3	4	5
	F28	Mean	**3.3287E + 03**	3.4277*E* + 03	3.3626*E* + 03	3.3302*E* + 03	3.3703*E* + 03
		Std	**1.7005E + 02**	1.7236*E* + 02	1.6371*E* + 02	1.0408*E* + 02	1.6007*E* + 02
		Rank	**1**	5	3	2	4
	F29	Mean	**3.3221E + 03**	3.3466*E* + 03	3.3369*E* + 03	3.3284*E* + 03	3.3642*E* + 03
		Std	**7.8055E + 01**	1.0081*E* + 02	9.4273*E* + 01	8.6562*E* + 01	1.0507*E* + 02
		Rank	**1**	4	3	2	5
	F30	Mean	**6.4195E + 05**	8.8875*E* + 05	1.2359*E* + 06	7.2195*E* + 05	2.2614*E* + 06
		Std	**7.2364E + 05**	1.0667*E* + 06	1.3062*E* + 06	1.1924*E* + 06	5.0252*E* + 06
		Rank	**1**	3	4	2	5

Friedman mean rank			**1.7241**	3.2414	3.2414	2.9655	3.8276
Rank			**1**	3	3	2	5

The best results are marked in bold.

**Table 9:** Results for tension/compression spring design problem.

Algorithm	Optimum variables			Optimum weight
	*d*	*D*	*N*	
**ERHHO**	**0.054919**	**0.50031**	**5.2144**	**0.010886**
SMA	0.056026	0.532	4.6974	0.011184
WOA	0.056172	0.53628	4.6338	0.011225
SSA	0.05	0.340474	11.3674	0.011378
SCA	0.051349	0.39299	8.7762	0.011166
HHO	0.057482	0.57567	4.1079	0.011618
DHHO/M	0.05624	0.53828	4.6045	0.011244
HHOCM	0.055303	0.51118	5.0275	0.010987

The best results are marked in bold.

**Table 10:** Results for pressure vessel design problem.

Algorithm	Optimum variables				Optimum cost
	*T*_*s*_	*T*_*h*_	*R*	*L*	
**ERHHO**	**0.8128337**	**0.414164**	**44.19005**	**152.3373**	**5,907.41**
SMA	0.8498743	0.4168857	45.62804	137.3114	5,953.6101
WOA	0.7379761	0.5032129	40.31962	200	6,100.539
SSA	0.8724656	0.4266437	46.7582	126.3416	6,004.6857
SCA	0.6869396	0.3790506	40.36443	200	6,078.1605
HHO	0.8971188	0.4377937	47.79634	116.8499	6,055.0952
DHHO	0.8516057	0.3951695	44.15988	152.6637	5,997.743
HHOCM	0.850937	0.4147511	45.41652	139.4434	5,947.2608

The best results are marked in bold.

**Table 11:** Results for the three-bar truss design problem.

Algorithm	Optimum variables		Optimum cost
	*x*1	*x*2	
**ERHHO**	**0.78842**	**0.40811**	**263.8523**
SMA	0.79893	0.37727	264.1663
WOA	0.80697	0.35801	264.0902
**SSA**	**0.7884**	**0.40816**	**263.8523**
SCA	0.80167	0.37081	264.052
HHO	0.79595	0.38721	263.893
DHHO	0.78073	0.43031	263.897
HHOCM	0.79599	0.38709	263.8935

The best results are marked in bold.

**Table 12:** Results for the cantilever beam design problem.

Algorithm	Optimum variables					Optimum weight
	*x*1	*x*2	*x*3	*x*4	*x*5	
**ERHHO**	**6.0509**	**5.2639**	**4.514**	**3.4605**	**2.1878**	**1.3402**
SMA	5.984	5.3074	4.5136	3.4321	2.248	1.3407
WOA	6.5083	6.1653	4.679	3.1335	1.6882	1.3837
SSA	5.9772	5.3966	4.4619	3.4675	2.1753	1.3403
SCA	5.6445	5.9607	5.0894	3.0544	2.2917	1.3753
HHO	6.0578	5.6231	4.2325	3.4302	2.2035	1.3445
DHHO/M	5.6908	5.647	4.7009	3.3578	2.1859	1.3467
HHOCM	6.0932	5.2465	4.633	3.3748	2.1476	1.3413

The best results are marked in bold.

**Table 13:** Results for the speed reducer design problem.

Algorithm	Optimum variables							Optimum weight
	*x*1	*x*2	*x*3	*x*4	*x*5	*x*6	*x*7	
**ERHHO**	**3.4976**	**0.7**	**17**	**7.3**	**7.8**	**3.35006**	**5.28553**	**2,995.4374**
SMA	3.49767	0.7	17	7.3	7.8	3.35007	5.28554	2,995.4379
WOA	3.49441	0.7	17	8.10001	7.97957	3.35128	5.32567	3,033.2286
**SSA**	3.49762	0.7	17	7.37353	8.14154	3.35019	5.28555	3,003.6298
SCA	3.6	0.7	17	7.6079	7.98083	3.39127	5.30003	3,061.4356
HHO	3.52699	0.7	17	7.3	7.80055	3.3504	5.28416	3,007.2009
DHHO	3.49737	0.7	17	8.04541	7.8	3.35194	5.28554	3,002.6565
HHOCM	3.49777	0.7	17	7.48788	7.99086	3.35156	5.28524	3,001.7286

The best results are marked in bold.

## Data Availability

The data used to support the findings of this study are available from the corresponding author upon request.
